# Black tea extract prevents lipopolysaccharide-induced NF-κB signaling and attenuates dextran sulfate sodium-induced experimental colitis

**DOI:** 10.1186/1472-6882-11-91

**Published:** 2011-10-11

**Authors:** Young-A Song, Young-Lan Park, Kyu-Yeol Kim, Cho-Yun Chung, Gi-Hoon Lee, Dae-Ho Cho, Ho-Seok Ki, Kang-Jin Park, Sung-Bum Cho, Wan-Sik Lee, Nacksung Kim, Bong-Whan Ahn, Young-Eun Joo

**Affiliations:** 1 Department of Internal Medicine, Chonnam National University Medical School, Gwangju, Korea; 2 Department of Pharmacology, Chonnam National University Medical School, Gwangju, Korea; 3 Department of Biochemistry, Chonnam National University Medical School, Gwangju, Korea

**Keywords:** Black tea, NF-κB, Macrophage, Dextran sulfate sodium, Colon inflammation

## Abstract

**Background:**

Black tea has been shown to elicit anti-oxidant, anti-carcinogenic, anti-inflammatory and anti-mutagenic properties. In this study, we investigated the impact of black tea extract (BTE) on lipopolysaccharide (LPS)-induced NF-κB signaling in bone marrow derived-macrophages (BMM) and determined the therapeutic efficacy of this extract on colon inflammation.

**Methods:**

The effect of BTE on LPS-induced NF-κB signaling and pro-inflammatory gene expression was evaluated by RT-PCR, Western blotting, immunofluorescence and electrophoretic mobility shift assay (EMSA). The *in vivo *efficacy of BTE was assessed in mice with 3% dextran sulfate sodium (DSS)-induced colitis. The severity of colitis was measured by weight loss, colon length and histologic scores.

**Results:**

LPS-induced IL-12p40, IL-23p19, IL-6 and IL-1β mRNA expressions were inhibited by BTE. LPS-induced IκBα phosphorylation/degradation and nuclear translocation of NF-κB/p65 were blocked by BTE. BTE treatment blocked LPS-induced DNA-binding activity of NF-κB. BTE-fed, DSS-exposed mice showed the less weight loss, longer colon length and lower histologic score compared to control diet-fed, DSS-exposed mice. DSS-induced IκBα phosphorylation/degradation and phosphorylation of NF-κB/p65 were blocked by BTE. An increase of cleaved caspase-3 and poly (ADP-ribose) polymerase (PARP) in DSS-exposed mice was blocked by BTE.

**Conclusions:**

These results indicate that BTE attenuates colon inflammation through the blockage of NF-κB signaling and apoptosis in DSS-induced experimental colitis model.

## Background

A substantial body of evidence demonstrates that various naturally occurring and dietary compounds present significant anti-inflammatory effects. For this reason, they represent potential molecules for the development of new drugs, designed for treatment of various inflammatory disorders, including inflammatory bowel disease (IBD) [1,2]. However, limited scientific evidence regarding the effectiveness of naturally occurring and dietary compounds and mechanistic understanding of their actions has prevented their incorporation into the mainstream medicine.

Tea including black tea, green tea or oolong tea is the most common consumed beverage worldwide. About 80% of total world tea production is consumed as black tea. Black tea is derived from the leaves of *Camellia sinensis*, and is fully fermented and oxidized. Although polyphenols are the most significant group of tea components, the chemical compositions of green and black tea are different. The main phenolic components of green tea are catechins. During the fermentation and oxidation process in the production of black tea, the substantial proportions of catechins are converted to dimeric and oligomeric flavanols such as theaflavins and thearubigins by a polyphenol oxidase [3-6]. The major polyphenols of black tea extract (BTE) such as theaflavins and thearubigins have been shown to possess anti-inflammatory, anti-oxidative, anti-mutagenic and anti-carcinogenic in *in vitro *and *in vivo *studies. Dietary intake of black tea has been associated with a reduced incidence of developing atherosclerosis, coronary heart disease, and gastrointestinal tract, liver, prostate cancer [7-14]. However, the underlying mechanisms responsible for health benefits of black tea are largely unknown as compared with those of green tea.

The IBD such as Ulcerative colitis and Crohn's disease is a chronic and relapsing condition of the intestinal inflammation of unknown etiology. It has been proposed that IBD causes dysregulated mucosal immune response in the intestinal wall facilitated by defects in epithelial barrier function and activation of immune cells with excessive production of pro-inflammatory mediators such as IL-1β, IL-6, IL-12p40, IL-23p19, TNF-α and IFN-γ resulting in tissue injury [15-20]. NF-κB is a nuclear transcription factor that regulates the expression of genes encoding pro-inflammatory mediators that play a key part in inflammation related injury such as IBD [21-24]. IBD and experimental intestinal inflammation models including dextran sulfate sodium (DSS), trinitrobenzene sulfonic acid (TNBS)-induced colitis and IL-10 knockout mice are characterized by NF-κB activation and increased expression of pro-inflammatory NF-κB target genes [25,26]. Previously, black tea polyphenols such as theaflavin and thearubigin exerted beneficial effects in TNBS-induced colitis through the inhibition of NF-κB activation [13,14]. But until now, there are no data about the impact of black tea on DSS-induced experimental colitis.

In the present study, we examined the impact of BTE on lipopolysaccharide (LPS)-induced NF-κB signaling in bone marrow derived-macrophage (BMM) and DSS-induced experimental colitis.

## Methods

### Cell culture and treatment

Bone marrow cells were isolated from 5- to 8-week-old C57/Bl/6 mice (Samtako Science, Daejeon, Korea) as previously described [27]. Mice were sacrificed by cervical dislocation. Femora and tibiae were aseptically removed and dissected free of adherent soft tissue. The bone ends were cut, and the marrow cavity was flushed out into a petri dish by slowly injecting MEM-α medium (Hyclone, Loan, UT, USA) at one end of the bone using a sterile 21-gauge needle. The bone marrow suspension was carefully agitated with a plastic pasteur pipette to obtain a single cell suspension. Bone marrow cells were washed and depleted of RBC by hypotonic lysis using RBC lysing buffer (Sigma-Aldrich, St. Louis, MO, USA). After washing twice with PBS, the cells were suspended in MEM-α medium supplemented with 10% FBS and 50 units/ml penicillin, 50 μg/ml streptomycin (Gibco, Grand Island, NY, USA). The number of viable cells was determined with trypan blue (Gibco) and bone marrow cells were cultured on 10 cm^2 ^tissue culture dishes in total amount of 2 × 10^6 ^cells/dish. 10 ng/ml of mouse macrophage colony stimulating factor (M-CSF, BioSource, Camarillo, CA) was added to every 10 cm dish to differentiate BMM. On day 3, non-adherent cells were discarded and adherent cells (immature BMM) were suspended in fresh MEM-α with M-CSF and used in subsequent experiment. All of the cells were cultured at 37°C under a humidified atmosphere containing 5% CO_2_. LPS from *Escherichia coli *(serotype 0111:B4) was also purchased from Sigma-Aldrich and dissolved in sterile, pyrogen free phosphate-buffered saline (PBS). Cells were pretreated with various concentrations of BTE (0-200 μg/ml) after which they were stimulated with LPS (0.5-1 μg/ml) for times indicated (0-1 h). All animal protocols were approved by the Institutional Animal Care and Use Committee of the Chonnam National University Hospital, Gwangju, Korea.

### Immunofluorescence

The cells were plated on 8-chamber slide (Nunc. Rochester, NY, USA). The cells were exposed to LPS (1 μg/ml) for 10 min in the absence or presence of 100 μg/ml BTE-pretreatment. Then cells were washed with PBS and fixed with 4% formaldehyde in RT. Next, cells were permeabilized using phosphate-buffered saline (PBS) containing 0.25% Triton X-100 and blocked with PBS containing 1% BSA and 10% FBS. Cells were subjected to staining with polyclonal anti-p65 antibody (Santa Cruz, Avenue, CA) overnight at 4°C. p65 in cells was visualized with Alexa 488 (green) conjugated secondary antibody (Invitrogen). Coverslips were mounted in ProLong Gold antifade reagent containing DAPI (Invitrogen) and analyzed using fluorescent microscopy.

### Electrophoretic mobility shift assay (EMSA)

Nuclear proteins were prepared following the previously described [28]. The treated cells were washed twice with PBS and resuspended in lysis buffer (10 mM HEPES (pH7.9), 0.5 mM KCl, 1.5 mM MgCl_2_, 0.5 mM DTT, 0.2 mM PMSF, 0.1% NP40). Cells were left on ice for 5 min and centrifuged at 12,000 × g for 5 min. Resulting pellet was resuspended in high salt buffer (20 mM HEPES (pH 7.9), 25% Glycerol, 1.5 mM MgCl2, 0.8 M KCl, 0.2 mM EDTA, 0.5 mM DTT, 0.2 mM PMSF) and centrifuged at 12,000 × g for 20 min. The supernatant was collected as the nuclear extract and protein concentration was estimated using BCA™protein assay (Thermo). The nuclear extracts were stored at -70°C. EMSA was performed using the LightShift™ Chemiluminescent EMSA kit (Pierce, Rockford, IL, USA) according to the manufacturer's instructions. The reaction mixtures (10 μl) containing about 5 μg nuclear extracts were incubated with 10 fmol of the biotin-labeled double-stranded oligonucleotide probes (NF-κB/p65 oligonucleotides; 5'-CAT CGG AAA TTT CCG GAA ATT TCC GGA AAT TTC CGG C-3'/5'-GCC GGA AAT TTC TGG AAA TTT CCG GAA ATT TCC AT G-3') in reaction buffer for 20 min at room temperature. Samples were then run into a 5% nondenaturing polyacrylamide gel and transferred to Biodyne™ B Nylon membrane (Thermo) in 0.5 × TBE buffer. The biotin-labeled NF-κB/p65 probe was detected with a using the streptavidin-horseradish peroxidase conjugate and the chemiluminescent substrate.

### Animals and DSS-induced colitis

The mice (C57/Bl/6 background) were used between 10 and 12 weeks of age. The mice were maintained in standard housing cages in a specific pathogen free (SPF) environment and allowed to drink and feed ad libitum at all times. BTE was incorporated in standard laboratory chow AIN-76 in different amounts (weight-percentages: 0.2% BTE, 1% BTE) (Dae Han Biolink Co., Chungbuk, Korea). The BTE composition is as follows: oxidized polyphenols 20%, catechins 3-5%, protein 5-10%, carbohydrate 10-15%, caffeine 2.2-5.2%, potassium content < 10%, moisture content < 6%, mineral/ash content < 20%. Mice (6/group) were pre-fed BTE-chow (0.2%, 1%) or control chow (AIN-76) for 3 days (loading period) as described previously. After this time, mice were given 3% DSS (MP Biomedicals; Aurora, OH) in drinking water for an additional 6 days. Control mice were given water. Water consumption was comparable between the different groups. Similarly, chow consumption (control AIN76 and BTE) was comparable between DSS and water control groups, both before and during the induction of colitis. Mice were monitored daily for weight loss as well as signs of rectal bleeding (Hemoccult, Beckmann Coulter Inc; Fullerton, CA). At day 6 of DSS administration, mice were sacrificed, sections were taken from the distal, proximal colon and cecum for histological assessment of inflammation. Animal experiments were performed in accordance with the guidelines of the institutional Animal Care and Use Committee of the Chonnam National University Hospital, Gwangju, Korea.

### Sample collection and histological evaluation

Mice were sacrificed at designated time-points by cervical dislocation. The entire colon was dissected and flushed with ice-cold PBS. Sections of cecum, proximal, and distal colon were taken, fixed in 10% neutral-buffered formalin for 24 h at room temperature and embedded in paraffin to provide sections for histological evaluation. Severity of colitis was evaluated in Hematoxylin-Eosin-stained sections by two independent observers blinded to the experimental conditions. Histological sections were scored using a validated scoring system as described previously [29-31].

### Real-time reverse transcription-polymerase chain reaction (RT-PCR)

Total RNA was extracted by using TRIzol reagent (Invitrogen, Carlsbad, CA, USA) and following the standard protocol. Measuring the quantity and purity of total RNA were determined using Nanodrop reader. Subsequently, 1 μg total RNA was converted to first strand cDNA using MMLV reverse transtcriptase (Invitrogen) and RNAsin (Takara, Otsu, Shiga, Japan). cDNA was amplified using gene specific primers and Go taq. Polymerase (Promega, Madison, WI, USA). Sequences of primers were 5'-CCAGCTTCTTCATCAGGGAC-3'/5'-GTCCCTGATGAAGAAGCTGG-3' for IL-12p40, 5'-CTCAAGGACAACAGCCAGTTC-3'/5'-GGCACTAAGGGCTCAGTCAG-3' for IL-23p19, 5'-GGATACCACCCACAACAGACC-3'/5'-AATCAGAATTGCCATTGCAC-3' for IL-6, 5'-ATCACTCATTGTGGCTGTGG-3'/5'-GTCGTTGCTTGGTTCTCCT-3' for IL-1β, 5'-ACCACAGTCCATGCCATCAC-3'/5'-TCCACCACCCTGTTGCTGTA-3' for GAPDH.

### Western Blot analysis

The protein concentration of lysates was measured using Bio-Rad quantification assay (Bio-Rad Laboratories; Hercules, CA). Proteins (20 μg) were separated using 10% (13% for caspase analysis) SDS-PAGE and transferred to nitrocellulose membranes. Antibodies to cleaved caspases 3, cleaved poly (ADP-ribose) polymerase (PARP), IκBα, phospho-IκBα (Cell Signaling Technology Inc, Beverly, MA), phospho-p65 (Santa Cruz) and β-actin (ICN; Costa Mesa, CA) were used as described by the manufacturer Following washing three times with TBST, membranes were incubated with secondary HRP-conjugated anti-mouse IgG for 1 h. After washing, the blots were detected with chemiluminescence (ECL) HRP substrate (Millipore, Billerica, MA) by image reader (Ras-4000, Fujifilm, Tokyo, Japan).

### Statistical analysis

Data are expressed as means ± SD. Groups of data were analyzed using Kruskal-Wallis non-parametric test and if the result indicated statistical differences among groups, comparisons between groups were conducted using Mann-Whitney U test. In vitro experiments were conducted in triplicates; representative results are shown. For in vitro experiments, data were analyzed by non-parametric *t*-test or Wilcoxon rank sum test where appropriate. A *p*-value of less than 0.05 was considered statistically significant.

## Results

### Effect of BTE on LPS-induced pro-inflammatory mediators expression in BMM

We investigated whether BTE could inhibit the LPS-induced pro-inflammatory mediators in BMM. The cells were pretreated with various concentrations of BTE (0-200 μg/ml) after which they were stimulated with 1 μg/ml of LPS for time indicated (1 h). BTE significantly reduced the LPS-induced IL-12p40, IL-23p19, IL-6, and IL-1β mRNA accumulations in various concentrations as determined by RT-PCR and densitometry (Figure 1A). The cells were pretreated with 100 μg/ml BTE for 1 h prior to different incubation times (1 or 4 h) with stimulation of 1 μg/ml LPS. BTE significantly reduced the LPS-induced IL-12p40, IL-23p19, IL-6, and IL-1β mRNA accumulations for different incubation times as determined by RT-PCR and densitometry (Figure 1B).

**Figure 1:** **Effect of BTE on expression of LPS-induced pro-inflammatory mediators in BMM**. RNA was isolated using TRIzol procedure, and 1 μg of total RNA was reverse transcribed and amplified using specific primer for IL-12p40, IL-23p19, IL-6, IL-1β and GAPDH. Band intensities were quantified by densitometry. Results are representative of 3 independent experiments. (A) The cells were pretreated with various concentrations of BTE (0-200 μg/ml) after which they were stimulated with 1 μg/ml of LPS for time indicated (1 h). BTE significantly reduced the LPS-induced IL-12p40, IL-23p19, IL-6, and IL-1β mRNA accumulations in various concentrations as determined by RT-PCR and densitometry. (B) The cells were pretreated with 100 μg/ml BTE for 1 h prior to different incubation times (1 or 4 h) with stimulation of 1 μg/ml LPS. BTE significantly reduced the LPS-induced IL-12p40, IL-23p19, IL-6, and IL-1β mRNA accumulations for different incubation times as determined by RT-PCR and densitometry.

### BTE inhibits LPS-induced IκBα phosphorylation/degradation, nuclear translocation of NF-κB/p65 and NF-κB DNA-binding activity in BMM

NF-κB regulates the production of pro-inflammatory mediators in cellular inflammation. To determine whether the inhibitory action of BTE on expression of pro-inflammatory mediators, was mediated through the inhibition of NF-κB signaling, we examined the cytoplasmic levels of IκBα and phospho-IκBα proteins by Western blotting. After 10, 30 min stimulation of BMM with LPS, the cytosolic IκBα protein was significantly phosphorylated and degraded. The LPS-induced IκBα phosphorylation/degradation was dramatically inhibited by coincubation LPS plus BTE (Figure 2A). The nuclear translocation of NF-κB/p65 follows IκBα phosphorylation/degradation. So, we tested if BTE perturbed the distribution of NF-κB/p65 as assessed by nuclear accumulation. As shown in Figure 2B, coincubation with LPS plus BTE inhibited the nuclear translocation of NF-κB/p65. Lastly, an EMSA on nuclear extracts of BMM by using a consensus oligonucleotide for NF-κB binding was performed. The induction of specific NF-κB binding with NF-κB site by LPS was markedly inhibited by coincubation with BTE (Figure 2C). These results suggested that inhibition of pro-inflammatory mediators production by BTE occurred via blocking of NF-κB signaling.

**Figure 2:** **Effect of BTE on LPS-induced NF-κB signaling in BMM**. The cells were pretreated with BTE (100 μg/ml) and then stimulated with LPS (1 μg/ml) for times indicated. (A) IκBα phosphorylation/degradation was evaluated by Western blotting. The LPS-induced IκBα phosphorylation/degradation was dramatically inhibited by coincubation LPS plus BTE. (B) Nuclear translocation of NF-κB/p65 was visualized by immunofluorescence. Coincubation with LPS plus BTE inhibited the nuclear translocation of NF-κB/p65. (C) An EMSA on nuclear extracts of BMM by using a consensus oligonucleotide for NF-κB binding was performed. BTE inhibited LPS-induced NF-κB DNA-binding activity. Bars represent the mean ± SD from three different experiments. (*p < 0.05, compared to unstimulated cells; #p < 0.05, compared to LPS stimulation). BTE, black tea extract; BMM, bone marrow-derived macrophage.

### BTE treatment attenuates DSS-induced experimental colitis

To test the therapeutic potential of BTE on intestinal inflammation, mice were pre-fed BTE-chow (0.2% and 1%) or control chow (AIN-76) for 3 days (loading period) and then exposed to 3% DSS in drinking water for an additional 6 days. Mice were monitored daily for clinical signs of disease that are manifested by weight loss, rectal bleeding and diarrhea. BTE-fed mice showed less significant weight loss than control diet-fed mice by day 4 (p < 0.05) (Figure 3). Mice were sacrificed at designated time points, the entire colon dissected and then directly imaged in a light imaging box. BTE-fed, DSS-exposed mice had significantly longer colons than control diet-fed, DSS-exposed mice (p < 0.05) (Figure 4A, B). Histological evaluation of the colon of BTE-fed, DSS-exposed mice indicated a significant decrease in colon inflammation compared to control diet-fed, DSS-exposed mice (p < 0.05) (Figure 5A, B).

**Figure 3:** **BTE attenuates DSS-induced experimental colitis as measured by weight loss**. Mice (6/group) were pre-fed BTE-chow (0.2%, 1%) or control chow (AIN-76) for 3 days (loading period). After this time, mice were given 3% DSS in drinking water for an additional 6 days. Weight loss in response to DSS is presented as percent of the starting weight (*p,0.05 versus control, #p,0.05 versus DSS alone). BTE-fed, DSS-exposed mice showed less significant weight loss than control diet-fed, DSS-exposed mice by day 6 (p < 0.05). Values are mean ± SEM; n = 6 in each group. BTE, black tea extract; DSS, dextran sulfate sodium.

**Figure 4:** **BTE attenuates DSS-induced experimental colitis as measured by colon length**. (A) Mice (6/group) were sacrificed at designated time points, the entire colon dissected and then directly imaged in a light imaging box. (B) BTE-fed, DSS-exposed mice had significantly longer colons than control diet-fed, DSS-exposed mice (*p < 0.05). BTE, black tea extract; DSS, dextran sulfate sodium.

**Figure 5:** **BTE attenuates DSS-induced experimental colitis as measured by histologic score**. (A) The proximal, distal colon and cecum of DSS-exposed mice were evaluated and coded sections were scored using a validated scoring system using a scale of 0 to 40 (*p < 0.05). Values are mean ± SD; n = 6 in each group. Histological evaluation of the colon of BTE-fed, DSS-exposed mice indicated a significant decrease in colon inflammation compared to control diet-fed, DSS-exposed mice (p < 0.05). (B) Representative histologic slides from control, DSS and 1% BTE+DSS groups (×200). DC, distal colon; PC, proximal colon; CE, cecum; BTE, black tea extract; DSS, dextran sulfate sodium.

### BTE treatment blocks NF-κB activation and apoptosis

We reasoned whether anti-inflammatory effect of BTE in response to DSS-induced injury is associated with blocking of NF-κB activity. Western blotting showed that DSS-induced IκBα phosphorylation/degradation and phosphorylation of NF-κB/p65 were blocked by BTE (Figure 6A, B). We next sought to investigate the impact of BTE on intestinal apoptosis following DSS-induced injury. An increase of cleaved caspase-3 and PARP in DSS-exposed mice was blocked by BTE treatment (Figure 6A, B). These findings indicate that BTE attenuates acute colon inflammation through blocking of NF-κB activation and apoptosis.

**Figure 6:** Effect of BTE on NF-κB signaling and apoptosis in DSS-induced experimental colitis. (A) Mice (6/group) were sacrificed after 6 (for total colon protein) days of 3% DSS exposure, respectively and protein (20 μg) was subjected to SDS-PAGE. IκBα, phospho-IκBα, phospho-p65, cleaved caspase 3, cleaved PARP and β-actin expression using specific antibodies respectively, and immunoreactive proteins were detected using the enhanced chemiluminescence (ECL) technique. DSS-induced IκBα phosphorylation/degradation and phosphorylation of NF-κB/p65 were blocked by BTE. An increase of cleaved caspase-3 and PARP in DSS-exposed mice was blocked by BTE treatment. (B) Band intensities were quantified by densitometry. Results are representative of 3 independent experiments. BTE, black tea extract; DSS, dextran sulfate sodium.

## Discussion

IBD is chronic relapsing intestinal inflammatory disorder. Although the etiology of IBD is currently unknown, converging evidence suggest that IBD results from aberrant innate immune responses to the enteric microbiota in genetically susceptible host [15-20]. Key participants in the innate immune response to the enteric microbiota are macrophages [18]. However, until now, the direct effects of BTE on bone marrow-derived macrophage (BMM) in intestinal inflammation have not been investigated. The production of pro-inflammatory mediators including inflammatory cytokines, chemokines and cell adhesion molecules is controlled by the activity of transcriptional factors, such as the nuclear factor-kappa B (NF-κB) in IBD. Thus, the activation of NF-κB is known to be extremely important in the pathogenesis of IBD and has been proposed as a major culprit and therapeutic target for IBD [21-24].

Previously, black tea polyphenol blocked NF-κB activity in various cell types including human lung adenocarcinoma cells and intestinal epithelial cells [8,32]. We first investigated the effect of BTE on expression of pro-inflammatory mediators and NF-κB signaling in LPS-stimulated BMM. Our study showed that BTE significantly reduced the LPS-induced IL-12p40, IL-23p19, IL-6, and IL-1β mRNA accumulations. Also, we observed that BTE prevented LPS-induced NF-κB activity in BMM through blockade of IκBα phosphorylation/degradation, decreased NF-κB/p65 nuclear translocation and DNA-binding activity of NF-κB. Therefore, BTE reduces the expression of pro-inflammatory mediators via the blockage of LPS-induced NF-κB signaling in BMM.

DSS, a sulfated polysaccharide administered to mice in drinking water, is directly cytotoxic to enterocytes of the basal crypts and leads to breakdown of intestinal barrier integrity, translocation of enteric microbiota, and induction of a colitis phenotype that is independent of the adaptive immune system. Therefore, the acute DSS-induced experimental colitis model is useful for study of innate immune mechanisms of colitis such as NF-κB and tissue repair [25,26]. Next, to assess the therapeutic efficacy of BTE on intestinal inflammation, mice were fed a BTE rich diet and then exposed to DSS. In our study, BTE-fed, DSS-exposed mice showed significantly less weight loss, longer colons and lower histologic score than control diet-fed, DSS-exposed mice. Eventually, BTE ameliorated the colon inflammation in DSS-induced experimental colitis model. We reasoned whether anti-inflammatory effect of BTE in response to DSS-induced injury is associated with blocking of NF-κB activity. Our study showed that DSS-induced IκBα phosphorylation/degradation and phosphorylation of NF-κB/p65 in colonic tissues were blocked by BTE. Recent studies showed that black tea polyphenols including theaflavin and thearubigin exerted protective effects in TNBS-induced colitis model and inhibited production of inflammatory mediators through the inhibition of NF-κB activation [13,14]. These and our results suggest that black tea have beneficial effects in various experimental colitis models and may be used to modulate inflammatory processes in IBD.

BTE, used in our study contains numerous chemical components including polyphenols, catechins, proteins, carbohydrate, amino acids, caffeine and so on. Our study has not directly identified the active ingredients responsible for these beneficial effects. BTE-mediated inhibition of NF-κB activity was replicated using black tea polyphenol, theaflavin in previous our study [32]. The oxidized polyphenols including theaflavin and thearubigin are major components of BTE, used in our study. Therefore, black tea polyphenols are at least partially responsible for the inhibition of NF-κB activity in our *in vitro *and *in vivo *studies.

Apoptosis is an essential mechanism for physiological and pathological cell death. Balance of cell growth and apoptosis determines normal tissue homeostasis [33,34]. A key feature of intestinal homeostasis is the host's ability to maintain the integrity of the epithelium and promote repair mechanisms following various injury insults. Thus, we next sought to investigate the impact of BTE on intestinal apoptosis following DSS-induced injury. Caspase-3 and PARP are key enzymes and executors of apoptosis [33,34]. An increase of cleaved caspase-3 and PARP in DSS-exposed mice was blocked by BTE treatment, leading to the inhibition of apoptosis.

## Conclusion

BTE treatment blocked the production of LPS-induced pro-inflammatory mediators and NF-κB activation in BMM. BTE treatment attenuated colon inflammation and inhibited NF-κB activation and apoptosis in DSS-induced experimental colitis. Therefore, BTE attenuates colon inflammation through the blocking of NF-κB signaling and apoptosis in DSS-induced experimental colitis model.

## Competing interests

The authors declare that they have no competing interests.

## Authors' contributions

YAS, YLP, KYK and CYC carried out the study and designed the experiments. GHL, DHC, HSK and KJP contributed reagents/materials/analysis tools. SBC and WSL analyzed data. NK and BWA supervised work and corrected the manuscript. YEJ conceived and designed experiments and wrote the manuscript. All authors read and approved the final manuscript.

## Pre-publication history

The pre-publication history for this paper can be accessed here:

http://www.biomedcentral.com/1472-6882/11/91/prepub
